# Mitochondrial-Targeted Antioxidant Peptide SS31 Prevents RPE Cell Death under Oxidative Stress

**DOI:** 10.1155/2022/6180349

**Published:** 2022-05-27

**Authors:** Yuan He, Zejun Chen, Ruixue Zhang, Zhuoya Quan, Yun Xu, Beilei He, Yuan Ren

**Affiliations:** ^1^Department of Ophthalmology, The Second Affiliated Hospital of Xi'an Medical University, Xi'an, China; ^2^Xi'an Medical University, Xi'an, China

## Abstract

This work aims at investigating the protective effects of the mitochondria-targeted peptide SS31, on mitochondria function, preventing human retinal pigment epithelial cell-19 (ARPE-19) cell apoptosis. The ARPE-19 cells were subjected to 24 h of intervention with H_2_O_2_ of various concentrations (0, 100, 150, 200, 250, 300, and 500 *μ*mol/L). Various concentrations of SS31 (10 nM, 100 nM, and 1 *μ*mol/L) pretreated the cells for 2 h. The MTT assay determined cell viability. ARPE-19 cell apoptosis was observed by 4′,6-diamidino-2-phenylindole (DAPI) staining under fluorescence microscope and detected by Annexin-V/PI staining under flow cytometry. The measurement of reactive oxygen species (ROS) release level used MitoSOX Red (a mitochondrial superoxide indicator) and the probe 2′-7′dichlorofluorescin diacetate (DCFH-DA). And with the use of a JC-1 probe, the mitochondrial membrane potential (MMP; ΔΨ*m*) was analyzed. Reverse transcription polymerase chain reaction (RT-PCR) and real-time PCR were responsible for measuring the levels of apoptosis related genes (Bcl-2, Bax, and Caspase-3). The cell viability increased significantly with SS31 pretreated (*P* < 0.05). In the SS31 + H_2_O_2_ group, the fluorescence of the cell nuclei with DAPI staining was weaker than H_2_O_2_ along group accordance with the decreased ratio of apoptotic cells (*P* < 0.05). The ROS generation decreased in SS31 pretreated group, with the increased ΔΨ*m*. The RT-PCR result showed decreased Bax gene and Caspase-3 gene expression with SS31 pretreatment, while increased antiapoptotic gene Bcl-2 (*P* < 0.05). We provide evidence that SS31 promotes resilience of RPE cells to oxidative stress by stabilizing mitochondrial function.

## 1. Introduction

Age-related macular degeneration (AMD) bears the major responsibility for progressive and irreversible central vision loss among the aged [1]. The most common characteristics of AMD are the formation of drusen and the alterations of RPE. The etiology of AMD is very complex, and the pathogenesis is having not been fully defined. Current research suggests a close connection between the oxidative damage of RPE cells and the pathogenesis of AMD, and the important cause of AMD is the dysfunction and metabolic abnormalities of RPE cells caused by oxidative damage of mitochondria [2]. Reactive oxygen species (ROS) are the main factor causing oxidative stress of RPE cells in retinal tissue. ARPE-19 is a spontaneously formed retinal pigment epithelial cell line. It is one of the cell models and tools commonly used by scientists that study vision. At present, it is mainly used to study the occurrence of ADM, the mechanism of disease or drug molecules with therapeutic activity, and to decipher cellular signal transduction events.

In addition to the traditional treatments, there are currently some studies on the treatment of AMD with antioxidants [3]. SS31 is a mitochondrial-targeted peptide synthesized by Peter W. Schiller and Hazel H. Szeto with 639.8 Da [4]. The polypeptide contains an alternating aromatic cation motif so that it can freely penetrate the cell membrane and be selectively concentrated on the inner membrane of the mitochondria without saturation. By targeting the mitochondria, it can clear ROS and inhibit lipid peroxidation. SS31 can reduce ROS generation both under physiological and pathological conditions. In addition, SS31 plays a variety of biological effects, such as inhibiting the transition of mitochondria membrane potential and mitochondria swelling, thereby preventing the release of CytC induced by Ca2^+^, etc., which can effectively reduce the cell apoptosis [5, 6].

The critical protective role of SS31 in some neurodegenerative diseases, such as ischemic brain injury, ischemia-reperfusion injury, and other diseases, has been repeatedly confirmed [7–9]. Researcher reported that SS31 is essential in resisting hippocampal neuron withering by downregulating Bax gene and protein expression and upregulating Bcl-2 gene expression in the Alzheimer's disease model [10–12]. SS31 also promotes electron transport and ATP synthesis in the mitochondrial inner membrane [9, 13, 14]. Preliminary studies in the treatment of diseases in ophthalmology have shown that SS31 can protect human lens epithelial cells by reducing oxidative damage to mitochondria [15] and 661 W mouse retinal photoreceptor cell lines [16]. In recent years, SS31 and other mitochondrial targeted peptides as a new type of antioxidant protective agent show a potent role on the neurodegenerative diseases [17, 18].

In this study, hydrogen peroxide (H_2_O_2_) was used on ARPE-19 cells to simulate the pathological process of AMD. We detected the protective effects of mitochondrial-targeted peptide SS31 on ARPE-19 cells under oxidative damage through cell viability and morphology observation, apoptosis, and the mitochondrial function detection. We speculated the possible new strategies for preventing and treating AMD from the mitochondrial-targeted antioxidant pathway.

## 2. Methods

### 2.1. Cells and Cell Cultivation

ARPE-19 cells, supplied by the American Type Culture Collection (ATCC, Rockville, MD), were cultivated in the medium and conditions as follows: medium: Dulbecco′s modified Eagle′s medium (DMEM) (Gibco, Grand Island, NY) + 10%fetal bovine serum (FBS) (Gibco, Grand Island, NY); culture conditions: 37°C, 5% CO_2_, and humidified atmosphere [19]. Cells were processed for the following assays when 75-80% confluence was observed.

### 2.2. Cell Viability

To detect ARPE-19 cell viability under oxidative stress (OS), cells were seeded into the wells of 96-well plates and treated with hydrogen peroxide (0, 100, 150, 200, 250, 300, and 500 *μ*mol/L), with or without 2 h pretreatment of SS31 (10 nM, 100 nM, and 1 *μ*M) for 24 h, followed by cultivation with DMEM (serum-free). Following MTT solution removal 4 h later, dimethyl sulfoxide (0.1 ml/well) was added to the plates, which were then shaken at ambient temperature for 10 min. A microplate spectrophotometer was utilized to read the absorbance_490 nm_ of the supernatant.

### 2.3. Cellular Morphology

After planting ARPE-19 cells into the wells of 6-well plates, they were treated with H_2_O_2_ (0, 100, 200, or 400 *μ*mol/L) alone or with 2 h pretreatment with SS31 (10 or 100 nmol/L or 1 *μ*mol/L) for 24 h. Then, observation of cellular morphology was performed with an inverted phase-contrast microscope (Leica, Frankfurt, Germany).

### 2.4. Determination of Cell Apoptosis Using 4′,6-Diamidino-2-phenylindole (DAPI Staining)

Nuclei morphology and cell apoptosis were determined by DAPI staining. After seeding ARPE-19 cells into the wells of 6-well plates, they were intervened by 200 *μ*mol/L of H_2_O_2_ at 37°C for 24 h, with or without 2 h of pretreatment with 1 *μ*mol/L SS31. They were then treated with two phosphate-buffered saline (PBS) rinsing and the subsequent 10 min of light tight cultivation with DAPI (5 *μ*g/ml). Afterward, PBS (Gibco, Grand Island, NY) was used to rinse each sample three times. Cell apoptosis was indicated the nucleus was fragmented or condensed. Observation of nuclei morphology and apoptosis alterations was performed with a fluorescence microscope manufactured by Leica, Frankfurt, Germany.

### 2.5. Determination of Cell Apoptosis Using Flow Cytometry (FCM)

The existence of apoptotic cells was evaluated by early changes of cell-related membrane phospholipid asymmetry in the early stage of apoptosis. Membrane cell phospholipid asymmetry loss is accompanied by exposure to phosphatidylserine. An Annexin-V (AV)/propidium iodide (PI) kit from KeyGEN BioTECH, Jiangsu, China was used for the determination of apoptosis. The ARPE-19 cells were treated with 200 *μ*mol/L for 24 h, alone or with the pretreatment of 1 *μ*mol/L SS31 for 2 h. 1 × 10^6^ cells/ml cells were then gathered for two PBS washes. Five hundred microliters of Binding Buffer was used to resuspend cells, after which 5 *μ*L each of AV and PI was placed into the cell suspension. Then came 15 min of cell incubation in the dark at ambient temperature. Finally, the samples were evaluated using FCM (BD Accuri, Franklin Lakes, New Jersey).

### 2.6. ROS Detection

In ARPE-19 cells, the ROS was evaluated by observation under fluorescence microscope using MitoSOX Red (KeyGEN BioTECH. Nanjing, Jiangsu, China) and FCM using 2′-7′dichlorofluorescin diacetate (DCFH-DA) probe. After seeding the cells into 6-well plates, they were intervened by H_2_O_2_ (200 *μ*mol/L) for 4 h at 37°C, with or without the pretreatment of 1 *μ*mol of LSS31 for 2 h. First, the ARPE-19 cells were rinsed once with PBS. Second, 1 *μ*L of MitoSOX Red was dissolved in 999 *μ*L of Hank's Balanced Salt Solution (HBSS) to make a concentration MitoSOX Red solution in every well. After shaking the plate lightly, the ARPE-19 cells were subjected to light tight incubation (37°C, 10 min). After light rinsing with warm buffer, they were observed by fluorescence microscope. Meanwhile, intracellular ROS in ARPE-19 cells was evaluated with DCFH-DA probe (KeyGEN BioTECH. Nanjing, Jiangsu, China). Cells were collected and suspended in DMEM containing 10 *μ*mol/L DCFH-DA, cultivated at 37°C for 20 min in dark, and mixed every 3-5 min. The samples were treated with three DMEM rinses for complete removal of DCFH-DA that did not enter ARPE-19 cells and then analyzed immediately using FCM. Setting parameters: Ex = 488 nm, and Em = 525 nm.

### 2.7. ΔΨ*m* Detection

As a ΔΨ*m* parameter, JC-1, a lipophilic dye that can permeate plasma and mitochondrial membranes, was used to detect ΔΨ*m* changes in cells. The dye, which glows red when it agglomerates in normal healthy cells with high mitochondria membrane potential, shows green fluorescence in those with low ΔΨ*m*. After seeding cells into the wells of 6-well plates, they were intervened by 200 *μ*mol/L H_2_O_2_ for 4 h at 37°C, with or without the pretreatment of 1 *μ*mol/LSS31 for 2 h. The JC-1 dye (YEASEN, Shanghai, China) was added to cells adjusted to 1 × 10^6^ cells/ml in 6-well plates in each sample. Then, the cells were treated with light tight incubation (37°C, 20 min), and the subsequent two rinses in particular buffer for immediate FCM analysis. Setting parameters: Ex = 488 nm; Em = 530 nm.

### 2.8. Reverse Transcription Polymerase Chain Reaction (RT-PCR)

After isolating from ARPE-19 cells using a kit (Thermo Fisher Scientific), the total RNA was synthesized into cDNA with another kit (Thermo Fisher Scientific). RNA yield (A260/A280) was spectrophotometrically monitored. RT was performed with the use of a First Strand cDNA Synthesis kit, and 2 *μ*g of RNA was incubated with the following items: oligo (dT) primer (1 *μ*l), 5X reaction buffer (4 *μ*l), RNase-free dH_2_O (7 *μ*l), 10 mM dNTP mix (2 *μ*l), Revert Aid RT (1 *μ*l), Ribo Lock RNase inhibitor (1 *μ*l), and RNase-free dH_2_O, in a final volume of 20 *μ*l. Reaction conditions of the mixture was as follows: 70°C for 5 min, followed by 37°C for 5 min and then 42°C for 60 min, and finally 70°C for 10 min. RT-PCR: cDNA (2 *μ*l), Taq PCR Master Mix (12.5 *μ*l), sense and antisense primers (1 *μ*l each), and dH_2_O, in a final volume of 25 *μ*l following the manufacturer's protocol, for 35 cycles. The thermocycling conditions used for RT-PCR were as follows: 35 cycles at 94°C, 60°C, and 72°C, all for 30 secs. After that, 1% agarose (agarose-to-TAE buffer solution: 1 g: 100 ml) was made and dissolved in a TAE buffer via microwave heating. Then, it was cool about 50°C and added with 5 *μ*l of ethidium bromide. The final RT-PCR product samples underwent electrophoresis. Finally, gel was imaged and analyzed.

### 2.9. Real-Time PCR

The RNA was isolated from ARPE-19 cells using the kit. QPCR was performed using a three-step amplifying protocol using PCR Master (Thermo Fisher Scientific). Mixes, as well as Real-time PCR Master Mixes (12.5 *μ*l), template cDNA (1,000 ng), and sense and antisense primers (0.5 *μ*l each), were diluted in a 20 *μ*l reaction volume. Reaction conditions: 95°C/10 min; followed by 40 cycles of 95°C/15 secs., 60°C/30 secs., 72°C/32 secs.; and finally 95°C/15 secs., 60°C/60 secs, and 95°C/15 secs. Each sample was repeatedly tested three times and quantification of expression levels used the 2-*ΔΔ*Ct method.

### 2.10. Statistical Processing

Data were statistically analyzed via SPSS *v*19.0 (SPSS, Chicago, IL). All analyses were performed independently at least three times. A one-way analysis of variance was adopted to test the collected data recorded as mean ± standard error of the mean, with *P* < 0.05 as the significance level.

## 3. Results

### 3.1. SS31 Inhibits Oxidative Damage-Induced ARPE-19 Cell Viability Decline

ARPE-19 cell viability was dose-dependently reduced in H_2_O_2_ treatment group (*P* < 0.05). Cell survival rate was reduced by 60% with 200 *μ*mol/L H_2_O_2_ (65% ± 3.04) versus the control group (95% ± 5.5), as shown in Figure 1(a). While pretreatment with SS31 gave rise to increased cell survival as compared to the H_2_O_2_ group (67% ± 3.9), followed by (71.9% ± 5.4), (76.4% ± 3.3), and (82.2% ± 3.4) (*P* < 0.05), and 1 *μ*mol/L SS31 was most obvious, as shown in Figure 1(b). From the statistical analysis data, SS31 showed no obvious side effect on ARPE-19 cell viability, with no notable difference found between control (89.3% ± 4.1) and SS31 (86% ± 4.0) groups (*P* < 0.05).

### 3.2. SS31 Morphologically Protects ARPE-19 against H_2_O_2_-Induced Cell Apoptosis

The number of living cells decreased as H_2_O_2_ concentration increased. As shown in Figure 2(a), ARPE-19 cells wizened gradually in morphology versus the control. By contrast, the number of living cells increased as the SS31 concentration increased, with cells tending to be normal in morphology gradually, as shown in Figure 2(b).

### 3.3. SS31 Prevents Cell Apoptosis in ARPE-19 Cells

DAPI staining showed concentrated nuclear chromatin and enhanced fluorescence of apoptotic cells. ARPE-19 cells with 24 h of 200 *μ*mol/L H_2_O_2_ exposure showed obvious apoptotic properties like concentrated chromatin and enhanced fluorescence. In contrast, the nuclear fluorescence was weak in control and SS31 groups. Pretreatment of SS31 attenuated fluorescence obviously, suggesting the protective role of SS31 towards ARPE-19 cells against oxidative damage (×200), as shown in Figure 3(a). PI and AV-negative (-) cells were considered live cells (bottom left); PI (-) while AV-positive (+) cells were viable apoptotic cells (bottom right); those with PI (+) and AV (+) were primarily nonviable apoptotic cells (top right); and those with PI (+) and AV (-) were nonviable nonapoptotic cells (top left). An evident increase of AV-positive ARPE-19 cells was observed after 24 h of H_2_O_2_ treatment. By contrast, 1 *μ*mol/L of SS31 (28.0%) was highly protective of ARPE-19 against H_2_O_2_ (37.7%), as shown in Figure 3(b). Obviously, SS31 showed no effect on cells alone (*P* < 0.05). A significant difference was present between control and H_2_O_2_ groups, as well as between SS31 + H_2_O_2_ and H_2_O_2_ groups (*P* < 0.05), as shown in Figure 3(c).

### 3.4. SS31 Significantly Reduces Mitochondrial ROS

MitoSOX red and DCFH-DA probe were applied to detect the ROS release level in ARPE-19 cells. The control cells showed weak red fluorescence. The red fluorescence intensity was significantly enhanced in H_2_O_2_ group, indicating that the release level of ROS was significantly increased. After the pretreatment of SS31, cell fluorescence intensity in this group dropped notably compared with H_2_O_2_ group. SS31 group and control group differed insignificantly in fluorescence intensity, as shown in Figure 4(a). Meanwhile, H_2_O_2_ group showed significantly stronger cell fluorescence intensity than control group, as indicated by the FCM diagram. After the pretreatment of SS31, the fluorescence intensity was statistically weaker versus the H_2_O_2_ group, indicating significantly reduced ROS release level (*P* < 0.05), as shown in Figures 4(b) and 4(c).

### 3.5. SS31 Elevates ΔΨ*m* under OS

For the purpose of determining the mitochondrial-mediated pathway in cellular disfunction and apoptosis under OS, the present study measured ΔΨ*m* using membrane potential indicator JC-1 by FCM. The image showed statistically reduced ΔΨ*m* of ARPE-19 cells under H_2_O_2_ treatment and increased number of cells with low membrane potential. Compared with the H_2_O_2_ group, the proportion of low mitochondrial potential of ARPE-19 cells in the 1 *μ*M of SS31 + H_2_O_2_ group was reduced (*P* < 0.05). The proportion of low mitochondrial membrane potential cells was not statistically different between SS31 and control groups (*P* < 0.05), as shown in Figures 5(a) and 5(b).

### 3.6. SS31 Regulates the Expression and mRNA Level of Apoptosis-Associated Genes

OS-induced apoptosis was also investigated by detecting apoptosis-associated gene expression. Administration of H_2_O_2_ was accompanied by notably enhanced expression and mRNA level of caspase-3 and Bax, both of which are linked to apoptosis, as well as suppressed Bcl-2, an antiapoptotic gene. However, the reverse was true under the intervention of SS31, namely, decreased caspase-3 and Bax levels and elevated antiapoptotic gene Bcl-2 level were observed, as shown in Figures 6(a) and 6(b).

## 4. Discussion

A large number of studies showed that abnormal changes in structure and dysfunction of RPE caused by oxidative damage is an important factor leading to AMD [19, 20]. In aging retinas, OS and ROS play a vital part in pathology [21]. Herein, ARPE-19 cell viability declined dose-dependently after exposure to H_2_O_2_, indicating that the cells were damaged in various degrees of OS. In this experiment, 200 *μ*mol/L of H_2_O_2_ was used to stimulate the cells for 24 h to establish the oxidative damage model of RPE during the pathogenesis of AMD. The viability of cells at this concentration is slightly greater than the half-lethal concentration, which was reasonable. In determining the concentration of SS31, this experiment was based on previous experimental studies [22]. Three concentrations of SS31 (10 nmol/L, 100 nmol/L, and 1 *μ*mol/L) were chosen for protecting the ARPE-19 cells. The cell viabilities in these concentrations were higher than that in the H_2_O_2_ group. According to the degree of increase, the optimal concentration of SS31 was 1 *μ*mol/L. At the same time, it was also found that when SS31 was used alone in ARPE-19 cells, it showed no toxicity to the cells.

Mitochondria are considered to be the starting site of endogenous apoptosis pathways and a key factor for cell survival and death. Mitochondria are critical in transduction process and expansion of death signals. Under the stimulation of apoptotic signals, the mitochondrial membrane potential decreases, ROS release level increases, permeability increases, and various apoptotic factors are released from the mitochondria into the cytoplasm, eventually leading to cell apoptosis [23, 24]. Typical morphological changes of apoptosis, such as chromatin condensation, cell shrinkage, and some organelles, ribosomes, and nuclear fragments, are wrapped by cell membranes to form apoptotic bodies. In this study, under the pretreatment of SS31, the number of apoptotic cells decreased, cell shrinkage was improved, and apoptosis was inhibited versus H_2_O_2_ group. In DAPI staining and FCM detection, the apoptosis rate of ARPE-19 cells after OS increased significantly, while SS31 can significantly reduce the apoptosis rate of cells.

Current research suggests that ROS is an important mediator of apoptosis, and it can act on various links in the mitochondrial apoptosis pathway. The signaling molecules in mitochondrial apoptosis also affect the generation of ROS. In this experiment, SS31 was shown to reduce the release level of ROS in ARPE-19 cells under OS. ROS release level was similar in SS31 and normal groups. It was preliminarily believed that SS31 can reduce the damage to retinal tissue under OS to a certain extent by reducing the release level of ROS.

In vitro experiments have confirmed that in the early stage of apoptosis, before the appearance of nuclear pathological changes, decrease of mitochondrial membrane potential is the manifestation of early cell apoptosis [25, 26]. In this experiment, after pretreatment of SS31, the green fluorescence was significantly weakened and the red fluorescence was enhanced, indicating a notably higher mitochondrial membrane potential than the H_2_O_2_ group, and SS31 had a certain protective effect against mitochondrial function and apoptosis in ARPE-19 cells. The mitochondrial membrane potential differed insignificantly between SS31 and control groups.

Recent evidence has shown the vital role of the mitochondrial pathway in the mechanism of cell survival. The caspase family and the Bcl-2 protein family currently received much attention among many apoptosis regulating genes. Of them, caspase-3 is the most crucial apoptotic executive protease in cell apoptosis, and the most important pair of apoptosis-regulating genes, which are opposite in function to each other, are the Bcl-2 gene and Bax gene [27]. Our research identified markedly elevated Bax and Caspase-3 expression and mRNA levels in ARPE-19 cells after cells were treated with H_2_O_2_, while decreased antiapoptotic gene Bcl-2, indicating that OS caused cell apoptosis. After the pretreatment of SS31, the results reversed, showing that SS31 plays a significant part in modulating apoptosis-related gene levels.

Previous studies have confirmed that SS31 can be detected in eye tissue after subcutaneous injection. Observation under confocal microscope and other methods confirmed that SS31 mainly enters the mitochondrial inner membrane after entering the cell [28]. In this experiment, SS31 shows no significant effect on mitochondrial function and apoptosis, and there was no cytotoxicity.

## 5. Conclusion

In our experiment, the protective actions of SS31 on ARPE-19 cells under OS were reported, which showed a potential value in treatment of AMD through enhanced RPE cell function. Since the molecular biological mechanism of SS31 was not studied in this experiment, genechip technology can be used to further explore SS31 in subsequent experiments.

## Figures and Tables

**Figure 1:** SS31 inhibits oxidative damage-induced ARPE-19 cell viability decline. (a) ARPE-19 cell viability reduced dose-dependently with increasing H_2_O_2_. (*n* = 9, ^∗^*P* < 0.05, vs. the control). (b) Impacts of different SS31 concentrations on cell viability under H_2_O_2_ concentration of 200 *μ*mol/L (*n* = 9, ^∗^*P* < 0.05, vs. the control). Data are indicated by mean ± SD.

**Figure 2:** SS31 protects ARPE-19 cells against OS in morphology. Observation under phase-contrast microscope. (a) ARPE-19 cell morphology under different H_2_O_2_ concentrations. (b) ARPE-19 cell morphology with different SS31 concentrations under H_2_O_2_ concentration of 200 *μ*mol/L (magnification, ×200).

**Figure 3:** SS31 inhibits ARPE-19 cell apoptosis. (a) ARPE-19 cell apoptosis detected by DAPI staining. Observation under fluorescence microscope (magnification, ×200). (b, c) Representative FCM images identified an obvious reduction in AV-positive cells in ARPE-19 cells pretreated with 1 *μ*mol/L of SS31, compared with those intervened by 24 h of H_2_O_2_. Quantitative analysis of AV-positive cells (*n* = 6, ^∗^*P* < 0.05 vs. the control; ^∗∗^*P* < 0.05 vs. the H_2_O_2_). Data are indicated by mean ± SD.

**Figure 4:** SS31 significantly reduces mitochondrial ROS. (a, b) Representative fluorescence images and FCM images of ARPE-19 cells, revealing an increased fluorescence in H_2_O_2_ group. Pretreatment with 1 *μ*mol/L SS31 significantly ameliorated the fluorescence (magnification, ×200). (c) Quantitative analysis (*n* = 6, ^∗^*P* < 0.05 vs. the control; ^∗∗^*P* < 0.05 vs. the H_2_O_2_). Data are indicated by mean ± SD.

**Figure 5:** SS31 increases ΔΨ*m* under OS. (a) After pretreatment with 1 *μ*mol/L of SS31, the ΔΨ*m* was increased compared with the H_2_O_2_ group. (b) Quantitative analysis of the percentage of cells with low mitochondrial membrane potential (*n* = 6, ^∗^*P* < 0.05 vs. the control. ^∗∗^*P* < 0.05 vs. the H_2_O_2_). Data are indicated by mean ± SD.

**Figure 6:** SS31 regulates the expression and mRNA levels of apoptosis-associated genes. (a, b) RT-PCR and real-time PCR results demonstrated that SS31 attenuated Bax and Caspase-3 gene expression and mRNA levels and improved the Bcl-2 gene (*n* = 6, ^∗^*P* < 0.05 vs. the control. ^∗∗^*P* < 0.05 vs. the H_2_O_2_). Data are indicated by mean ± SD.

## Data Availability

The datasets used and/or analyzed during the current study are available from the corresponding author on reasonable request.

## References

[1] Ong B. B., Ah-Fat F. G. (2016). Age-related macular degeneration. *British Journal of Hospital Medicine*.

[2] Khandhadia S., Lotery A. (2010). Oxidation and age-related macular degeneration: insights from molecular biology. *Expert Reviews in Molecular Medicine*.

[3] Wei Q.-Q., Yu J. (2017). Research advances in antioxidant treatment of age-related macular degeneration. Recent advances. *Ophthalmology*.

[4] Schiller P. W., Nguyen T. M., Berezowska I. (2000). Synthesis and in vitro opioid activity profiles of DALDA analogues. *European Journal of Medicinal Chemistry*.

[5] Szeto H. H. (2006). Mitochondria-targeted peptide antioxidants: novel neuroprotective agents. *The AAPS Journal*.

[6] Petri S., Kiaei M., Damiano M. (2006). Cell-permeable peptide antioxidants as a novel therapeutic approach in a mouse model of amyotrophic lateral sclerosis. *Journal of Neurochemistry*.

[7] Wu J., Zhang M., Hao S. J. (2015). Mitochondria-targeted peptide reverses mitochondrial dysfunction and cognitive deficits in sepsis-associated encephalopathy. *Molecular Neurobiology*.

[8] Stelmashook E. V., Isaev N. K., Genrikhs E. E., Novikova S. V. (2019). Mitochondria-targeted antioxidants as potential therapy for the treatment of traumatic brain injury. *Antioxidants*.

[9] Zhao W. Y., Han S., Zhang L., Zhu Y. H., Wang L. M., Zeng L. (2013). Mitochondria-targeted antioxidant peptide SS31 prevents hypoxia/reoxygenation-induced apoptosis by down-regulating p66Shc in renal tubular epithelial cells. *Cellular Physiology and Biochemistry*.

[10] Hao Z. H., Huang X., Wang M. R. (2017). SS31 ameliorates age-related activation of NF-*κ*B signaling in senile mice model, SAMP8. *Oncotarget*.

[11] Jia Y. L., Sun S. J., Chen J. H. (2016). SS31, a small molecule antioxidant peptide, attenuates *β*-amyloid elevation, mitochondrial/synaptic deterioration and cognitive deficit in SAMP8 mice. *Current Alzheimer Research*.

[12] Reddy P. H., Manczak M., Kandimalla R. (2017). Mitochondria-targeted small molecule SS31: a potential candidate for the treatment of Alzheimer's disease. *Human Molecular Genetics*.

[13] Birk A. V., Liu S., Soong Y. (2013). The mitochondrial-targeted compound SS-31 re-energizes ischemic mitochondria by interacting with cardiolipin. *Journal of the American Society of Nephrology*.

[14] Chakrabarti A. K., Feeney K., Abueg C. (2013). Rationale and design of the EMBRACE STEMI study: a phase 2a, randomized, double-blind, placebo-controlled trial to evaluate the safety, tolerability and efficacy of intravenous Bendavia on reperfusion injury in patients treated with standard therapy including primary percutaneous coronary intervention and stenting for ST-segment elevation myocardial infarction. *American Heart Journal*.

[15] Ma W., Zhu X., Ding X. (2015). Protective effects of SS31 on t-BHP induced oxidative damage in 661W cells. *Molecular Medicine Reports*.

[16] Pang Y., Wang C., Yu L. (2015). Mitochondria-targeted antioxidant SS-31 is a potential novel ophthalmic medication for neuroprotection in glaucoma. *Medical Hypothesis, Discovery and Innovation in Ophthalmology*.

[17] Babizhayev M. A. (2016). Generation of reactive oxygen species in the anterior eye segment. Synergistic codrugs of N-acetylcarnosine lubricant eye drops and mitochondria-targeted antioxidant act as a powerful therapeutic platform for the treatment of cataracts and primary open-angle glaucoma. *BBA Clinical*.

[18] He Y., Leung K. W., Ren Y., Pei J., Ge J., Tombran-Tink J. (2014). PEDF improves mitochondrial function in RPE cells during oxidative stress. *Investigative Ophthalmology & Visual Science*.

[19] Cao Y., Fang Y., Mu J., Liu X. (2016). High salt medium activates RhoA/ROCK and downregulates eNOS expression via the upregulation of ADMA. *Molecular Medicine Reports*.

[20] Shen J. K., Dong A., Hacktt S. F., Bell W. R., Green W. R., Campochiaro P. A. (2007). Oxidative damage in age-related macular degeneration. *Histology and Histopathology*.

[21] Yildirim Z., Ucqun N. I., Yildirim F. (2011). The role of oxidative stress and antioxidants in the pathogenesis of age-related macular degeneration. *Clinics*.

[22] Wang W., Liu X., Ren Y. (2019). PEDF protects human retinal pigment epithelial cells against oxidative stress via upregulation of UCP2 expression. *Molecular Medicine Reports*.

[23] Cai J., Yang J., Jones D. P. (1998). Mitochondrial control of apoptosis: the role of cytochrome _c_. *Biochimica et Biophysica Acta (BBA)-Bioenergetics*.

[24] Hengartner M. O. (2000). The biochemistry of apoptosis. *Nature*.

[25] Petit P. X., Lecoeur H., Zorn E., Dauguet C., Mignotte B., Gougeon M. L. (1995). Alterations in mitochondrial structure and function are early events of dexamethasone-induced thymocyte apoptosis. *The Journal of Cell Biology*.

[26] Zamzami N., Machetti P., Castedo M. (1996). Inhibitors of permeability transition interfere with the disruption of the mitochondrial transmembrane potential during apoptosis. *FEBS Letters*.

[27] Dong Y. J., Gao W. J. (2012). The role and relationship of bcl-2, bax and caspase-3 in apoptosis. *Chinese Journal of Gerontology*.

[28] Zhao K., Zhao G. M., Wu D. (2004). Cell-permeable peptide antioxidants targeted to inner mitochondrial membrane inhibit mitochondrial swelling, oxidative cell death, and reperfusion injury. *The Journal of Biological Chemistry*.

